RETRACTED

# Construction of a Basic Japanese Teaching Resource Base Based on a Deep Neural Network under a Big Data Environment

**DOI:** 10.1155/2022/4897660

**Published:** 2022-09-10

**Authors:** Yue Wang, Jianhua Ma, Tong Zhang

**Affiliations:** ^1^Changchun Normal University, Changchun 130032, China; ^2^Changchun Guanghua University, Changchun 130000, China

## Abstract

A challenge for education and teaching in universities is posed by “Internet plus,” which has made numerous educational resources at universities richer and more accessible. The development of a professional Japanese teaching resource base should be centered on the needs and characteristics of Japanese teaching in universities, as well as establish and enhance the mechanism for resource base construction. All forms of instructional resources should also continuously be updated and improved in order to realize the diversified, systematic, open, and long-term development of Japanese instructional resources. In light of the current state of the information technology industry's rapid expansion, this essay examines a few issues with the building of a Japanese teaching resource database. A fundamental Japanese teaching resource database built on DNN was created as a result. The CNN technology is used in this study to create the Arduino device identification application. Utilizing gadgets in the learning process, learners can obtain learning resources using the Arduino device identification program before engaging in learning activities. The experimental findings also demonstrate that the precision rate and recall rate of the Japanese teaching resource database system developed in this study may achieve about 93 and 94 percent, respectively. Its performance is better than the conventional teaching resource system, and it can offer top-notch teaching resources for teaching fundamental Japanese.

## 1. Introduction

In recent years, universities have actively improved and reformed information teaching, exploring the establishment of more efficient and convenient teaching forms that keep pace with the times and promoting the sharing of high-quality instructional resources. The informatization process of education has achieved fruitful results and improved the efficiency of teaching and management [1]. However, in the process of educational informatization, some problems have also appeared. Instructional resources have gradually exposed many disadvantages in design and application in practical application and promotion. One of the most difficult problems is that different application systems in universities have independent data, different system structures, and a lack of communication mechanisms, which leads to the emergence of many “information islands.” The design, development, and sharing of high-quality educational and instructional resources is one of the important tasks of educational informatization. At present, each school regards the construction of a professional teaching resource database as an important project to enhance connotation construction and realize information-based teaching. Under the condition of informatization, the resources of Japanese teaching will be richer and higher quality and will play a greater role after the interaction between online and offline [2]. In Japanese teaching, network resources will become technical support and learning resources for students. With the support of multimedia and computers, it is very convenient to obtain and use network resources. Using computers and multimedia can obtain information conveniently and quickly, which not only gives students various channels to learn Japanese but also enriches the materials and resources that can be applied in Japanese class and makes it easier for students to accept new knowledge [3]. The Japanese teaching resource pool sharing platform can collect scattered and isolated data and build it into an independent whole that is conducive to sharing, thus improving the efficiency and security of information services in universities [4]. This can not only improve the information teaching level of Japanese teaching but also stimulate students' interest in learning Japanese.

RETRACTED

The core purpose of a professional teaching resource database is to fully utilize the benefits of network resources, share resources, and establish a high-capacity, open, interactive, and information-based teaching service system with teaching content as the primary content that adapts to network development. In order to adapt to the information era, the creation of Japanese teaching resource databases is a new trend in school reform and a new type of Japanese teaching in universities [5]. The development of students' listening, speaking, reading, and writing skills is equally as important in Japanese instruction as it is in other languages, and this is likewise the main objective of Japanese instruction. Japanese language instruction, and basic Japanese instruction in particular, should go beyond the content of textbooks to include explanations of grammar, vocabulary, and other elements in conjunction with relatively recent social and cultural themes. This can not only liven up the classroom environment and inspire students' excitement for learning, but it can also teach pupils the most recent material, necessitating timely knowledge updates from qualified teachers [6]. The neural network of the human brain is represented by the abstract structure NN (neural network). To create an operational network, each neuron is linked to every other neuron in the layer below it. A convective neural network, or CNN for short, is a feedforward neural network with depth hierarchy and convolution calculation. It can learn audio, images, texts, etc. with little computational effort because of the sparse connections between CNN layers and the hidden layer's sharing mechanism for convolution kernel parameters. It does not need to do any additional data translation in order to mine its high-dimensional implicit features. In this research, DNN (Deep Neural Network) [7] is [8] introduced to the creation of teaching resource databases, and the creation of a basic Japanese teaching resource database based on DNN is studied. To make it easier for users to identify the instructional resources they need and to increase the utilization of Japanese educational resources. The following are the article's innovative points:

1. This article analyzes the requirements, theoretical underpinnings, users, characteristics of the content, and issues that should be taken into consideration when building a basic Japanese teaching resource database to improve the level of application of contemporary information technology and the autonomy of mobile network learning for Japanese learners and to create more high-quality basic Japanese instructional resources. The findings demonstrate that this methodology has the potential to significantly and successfully increase the rate at which Japanese instructional resources are used.
2. This paper develops the Arduino device identification program using CNN technology. Learners can use the Arduino device identification program to find learning materials related to devices during the learning process, then engage in learning. The creation of a Japanese teaching resource database has made it possible to publish, search for, and maintain educational materials. The platform implements the data integration function proposed in this paper and creates an operational model for seamless connection between various systems.

RETRACTED

## 2. Related Work

The emerging network technology, represented by the Internet and mobile Internet, is driving the traditional teaching mode, learning resources, and learning methods towards digitalization, networking, and intelligence, and driving the traditional paper-based teaching materials towards integration and three-dimensional development. The construction of a professional teaching resource database is imminent, and many scholars have studied it at present.

Wei designed an XML-based university teaching resource database-sharing platform system. In this system structure, XML is used as a data exchange format to solve the problem of shared data among heterogeneous systems, and the data of three existing systems in universities is integrated [9]. Zhe et al. pointed out that the professional teaching resource library is based on the realization of students' self-learning, with a friendly interface, clear sections, and simple and clear search; and can show the wisdom of front-line teachers and teaching achievements, with distinctive interactive learning characteristics of a higher vocational education platform [10]. Haugen F designed a teaching resource integration method based on CNN, including the design of a CNN-based Arduino device identification program and the construction of an Arduino device learning resource library [11]. Cousin M designed a new sharing model, which can decentralize resource storage but concentrate resource description on the premise of ensuring the normal operation of existing application systems. The resource management in this shared model should involve the participation of all subsystem users to make the management of data resources more convenient [12]. Lu et al. pointed out that in order to reduce the operation and management costs of the platform and resource library, teachers as the main personnel should continuously strengthen their platform management capabilities and master the basic skills of platform operation and management; have the ability to solve and supervise the day-to-day platform operation and resource library management [13]. Saito, in view of the common problems in education and teaching, combined with the technical advantages of two-dimensional code, analyzed the feasibility of the application of two-dimensional code in education and teaching. He believes that the application of two-dimensional codes in teaching is feasible and the effect is predictable [14]. Nakamichi pointed out that through learning in the information-based teaching platform and resource library, students can see richer grammar, sentences, etc. than in classroom teaching, so as to continuously improve students' ability to understand and apply knowledge [15]. Takeuchi professional teaching resource library fully considers the characteristics of students' learning and [16] cognition, etc., and follows the principle of “practical and sufficient.” According to the professional construction goals and the requirements of the talent training plan, fully explore the learners' interests, language learning, and occupational plans for helpful information to achieve the school's “knowledge + skills” talent training goal [17].

This paper highlights the necessity, theoretical foundation, users, content characteristics, and problems that should be taken into consideration in the construction of a basic Japanese teaching resource database from the perspective of concept discrimination, on the basis of a thorough analysis of concepts. It also examines a few issues to the creation of a database of Japanese teaching resources. On the basis of this, a fundamental DNN-based database of teaching resources for Japanese is built. In this study, CNN technology is used to create the Arduino device identification application. The Arduino device identification program enables learners to find learning materials about the devices used in the learning process before engaging in learning activities. The creation of a Japanese teaching resource database has made it possible to publish, search for, and manage educational materials. The platform implements the data integration function provided in this work and creates an operational model for seamless interaction between various systems.

RETRACTED

## 3. Methodology

### 3.1. DNN Technology Foundation

Deep learning has drawn the attention of more and more scholars in recent years as a brand-new discipline with rapid progress. Deep learning provides clear advantages in modeling and feature extraction over the shallow models of prior years. Deep learning, a novel technology in machine learning algorithm research, is descended from artificial neural network research [18]. Each neuron in the artificial neural network is connected to every other neuron in the adjacent layer to form an operating network, which is an abstraction of the neural network found in the human brain. The creation of a NN model requires no prior formula and can handle a variety of data types. Its benefits include strong nonlinear mapping capabilities, self-organization, self-adaptation, good fault tolerance, and self-learning capabilities. When dealing with complicated variables and connections, NN is particularly well suited for pattern recognition, data mining, and classification. CNN [19] is a feedforward NN with a depth hierarchy and convolution calculations. Because the connections between CNN levels are sparse and the hidden layer uses a sharing method for convolution kernel parameters, it can learn music, images, texts, and other types of data with little computational effort and mine its high-dimensional implicit features. The input data does not require any further conversion at the same time. Weight sharing, local connection, and pooling are some of CNN's features that successfully reduce the number of training parameters and the network's complexity. A multi-layer DNN typically has three layers: an input layer, a hidden layer, and an output layer. However, the layer-by-layer training method can address the issue that DNN is challenging to train to optimal performance. The structure of DNN is depicted in Figure 1.

RETRACTED

Convolution networks put a more efficient feature learning component on the foundation of multi-layer deep neural networks, giving them a higher capability for feature learning. In particular, the original full connection layer is inserted before the convolution layer and pool layer are connected via local displacement. The pooling layer lowers the resolution of feature surfaces in order to acquire spatially invariant features. Each neuron in the pooling layer pools the local receptive field in order to perform the second feature extraction function. The most notable distinction between CNN and shallow NN is the partial connection between neurons of two neighboring layers in CNN as opposed to a full connection in shallow NN. CNN is a type of deep NN, though, and so it will not experience the insurmountable issues that conventional shallow NN does. The use of CNN for small text has a positive impact on gathering local information. When recognizing images, we can move via sliding windows from left to right and up to down to detect local information. The most popular technique for modifying the parameter weight in a CNN model is the gradient descent method, which minimizes the loss function. The precision of the network is continually increased through thousands, and even tens of thousands, of repeated training sessions, layer by layer.

### 3.2. Basic Japanese Teaching Resource Library

Under the current information background, Japanese teachers will use multimedia technology to assist in teaching, and the use of information platforms and Japanese teaching resource databases can effectively save teachers' teaching time. For example, saving teachers' time to write Japanese blackboard writing will increase the time to explain more useful Japanese knowledge points to students in disguise. Some schools and teachers have made many attempts at teaching of network resources before, but due to various reasons, relevant personnel have not correctly recognized the real significance and value of the method of network resources in teaching practice [20]. This kind of network resource teaching, which lacks the guidance of molding theory, often gains little in teaching practice, and it is difficult to achieve the expected effect. The construction of a basic Japanese teaching resource database can enrich students' learning resources, provide a platform for students to collaborate and communicate, and increase students' autonomous learning. There are mainly three groups of people who use Japanese information platforms and Japanese teaching resource databases. The first group is the teachers. In the platform and resource database, teachers can choose and consult relevant teaching materials according to their own teaching needs and provide materials and information for their teaching. The design of instructional resources includes problem-solving strategies, implementation plans, or implementation strategies. In addition, the digital instructional resource should be designed with background analysis tools, which can be used to collect the data on learners' Japanese learning processes in time and form conclusive reflection to monitor or correct students' learning behavior. The construction of a basic Japanese teaching resource database can be divided into a spoken Japanese resource database, a Japanese listening resource database, a Japanese grammar and vocabulary resource database, a Japanese international ability test resource database, etc. According to the complexity of Japanese information instructional resources, the instructional resource can generally be divided into three categories: (1) Media resources, such as text, audio, and video, graphics, and images, animation. (2) Some simply made courseware, micro courses, online courses, and other resources. (3) Resources such as virtual simulation teaching software and online course platform developed by the system.

RETRACTED

The design of Japanese instructional resources should pay attention to language input and output from form to content, strengthen learners' skills training in Japanese listening and speaking by using mobile networks, and learn Japanese cultural knowledge through various resources [21]. The Japanese resource database should enable students to upload or download resources accurately, reduce the time for students to choose suitable resources, and facilitate students' ability to quickly and comprehensively find the learning information they need. By using the Japanese resource database, students can see several times more grammar examples than in class, and then improve their grammar comprehension and application ability. Network resources can effectively help students to learn independently. Teachers need to guide students purposefully, help students extend from the classroom to extracurricular activities, let students use network resources to acquire knowledge actively, and make students learn Japanese more flexibly. As the center and focus of Japanese learning, the ultimate goal of Japanese learning is that students can master test-related skills through learning. On this issue, Japanese teachers should consider using teaching methods related to network resources to explain knowledge points related to examinations in class. Japanese instructional resources are presented by multimedia embedding such as words, languages, animations, sounds, and images. There are problems in embedding video, microcases, microprojects, training, etc. Video explanation is more situational, which is conducive to stimulating students to participate in learning and promoting knowledge construction. The Japanese teaching resource database not only needs to publish and update various instructional resources regularly and timely after its completion, but more importantly, it needs to attract more students' attention and use the platform and resource database, which is the purpose of the platform and Japanese teaching resource database construction.

RETRACTED

### 3.3. Construction of Basic Japanese Teaching Resource Base Based on DNN

The overall construction goal of the Japanese teaching resource database is to fully utilize the benefits of the network, and provide all types of information including instructional resources for basic core courses of the Japanese major, Japanese exam question banks, professional qualification certification, and enterprise industry trends, etc., pay attention to the improvement of students' self-learning ability, and integrate employment information and interactive communication. The development of the fundamental Japanese teaching resource base was theoretically underpinned by constructivism learning theory. According to the constructivism philosophy, learning is a process of actively accumulating knowledge. Students with certain social and cultural backgrounds actively absorb and digest information by utilizing quality learning tools to create their cognitive structures. The creation of a platform interface is crucial for the development of a Japanese teaching resource database, which aims to actualize students' autonomy in learning. To create a learning platform with distinct educational qualities that can interact with one another, the resource pool should be clear and user-friendly, simple to use when looking for Japanese learning content, and clear when conducting searches. It should also be able to demonstrate the wisdom and teaching accomplishments of front-line Japanese teachers. The creation of high-quality digital basic Japanese instructional resources based on DNN is one of the goals of the construction of basic Japanese teaching resources, which also aims to raise the application level of modern information technology and foster independent learning among Japanese students. The foundational database of teaching materials in Japanese should be open, adaptable, interactive, useful, and scalable. The teaching resource database module can supply teachers and students with rich educational resources thanks to the aforementioned qualities, but it can also give them access to a larger learning environment. Students can fully utilize the teaching resource database's contents to increase their interest in studying Japanese. The properties of CNN are the basis for this paper's decision to use CNN to mine the data for an educational resource. For training and problem-solving in joint probability matrix decomposition models, implicit characteristic matrices that represent resources using CNN weight parameters are constructed. The primary function of the CNN framework is to extract implicit feature vectors from resources and mine their potential features from basic Japanese instructional materials. The identification of an Arduino device and model training process is shown in Figure 2.

RETRACTED

Cross entropy is a widely used loss function. This paper also uses cross entropy as the loss function. The formula of cross entropy is as follows:

(1) $$\begin{array}{c} H\left(p,q\right)=-\sum_{x}p\left(x\right)\log\;q\left(x\right). \end{array}$$

When it is used as the loss function of NN, *p* represents the correct answer and *q* represents the predicted value. The smaller the value of cross entropy, the closer the two probability distributions are, which means the better the constructed NN model. For all *m* samples, use the forward propagation algorithm to calculate the activation values of all neurons; for the *L* layer network, calculation is as follows:

(2) $$\begin{array}{c} \delta^{\left(L\right)}=\left[\begin{array}{c} \delta_{\left(1\right)}^{\left(4\right)}\\ \delta_{\left(2\right)}^{\left(4\right)}\\ \ldots \\ \delta_{\left(m\right)}^{\left(4\right)} \end{array}\right]\\ =\left[\begin{array}{c} -\left(y_{1}-{\hat{y}}_{1}\right)\sigma \prime \left(z_{0}{\;}_{\left(1\right)}^{\left(4\right)}\right)\\ -\left(y_{2}-{\hat{y}}_{2}\right)\sigma \prime \left(z_{0}{\;}_{\left(2\right)}^{\left(4\right)}\right)\\ \ldots \\ -\left(y_{m}-{\hat{y}}_{m}\right)\sigma \prime \left(z_{0}{\;}_{\left(m\right)}^{\left(4\right)}\right) \end{array}\right]. \end{array}$$

*l* starts from the *L* − 1 layer and decreases to 2, and calculates as follows:

(3) $$\begin{array}{c} \delta^{\left(l\right)}=\delta^{\left(l+1\right)}{\left(W^{\left(l\right)}\right)}^{T}\sigma \prime \left(z^{\left(l\right)}\right). \end{array}$$

Compute the partial derivatives of the error function with respect to the network parameters of each layer as follows:

(4) $$\begin{array}{c} \frac{\partial \text{Cost}}{\partial w^{\left(l\right)}}={\left(a^{\left(l\right)}\right)}^{T}\delta^{\left(l+1\right)},\;l=1,\ldots ,L-1. \end{array}$$

Using the gradient descent method, execute as follows:

(5) $$\begin{array}{c} W^{\left(l\right)}=W^{\left(l\right)}-\alpha \frac{\partial \text{Cost}}{\partial w^{\left(l\right)}},\;l=1,\ldots ,L-1. \end{array}$$

Calculate the error in accordance with the error function, then stop, if the error is less than the predetermined threshold or the iteration times exceed the predetermined threshold. The majority of the model developed in this paper is composed of five layers, including two convolution layers and three full connection layers. The output layer is the last complete connection layer. In the convolution layer, ReLU is used as the activation function. Each convolution layer is followed by a pool layer, which is pooled and locally normalised. The output layer's full connection layer, which is the last layer, employs the Softmax regression model. The test question is represented as a dense digital matrix *T*_*j*_ ∈ *R*^*p*×*l*^ by connecting the word vectors in the test question information, as shown in the following formula:

(6) $$\begin{array}{c} T_{j}=\left[\ldots ,w_{i-1},w_{i},w_{i+1},\ldots \right]. \end{array}$$

Among them, *p* is the dimension of the vector; *l* represents the number of word vectors. A test item context feature *c*_*i*_^*j*^ ∈ *R* is extracted by the *j* th shared weight *W*_*c*_^*j*^ ∈ *R*^*p*×*ω*^, and its window size *ω* represents the number of surrounding words, which satisfies the following equation:

(7) $$\begin{array}{c} c_{i}^{j}=\text{fun}\left(W_{c}^{j}⊗D_{\left(:i:\left(i+\omega -1\right)\right)}+b_{c}^{j}\right). \end{array}$$

Among them, “⊗” represents the convolution operation, *b*_*c*_^*j*^ ∈ *R* is the deviation corresponding to *W*_*c*_^*j*^; fun is a nonlinear excitation function. This paper uses ReLU to avoid the vanishing gradient problem. Then, the context feature vector *c*^*j*^ ∈ *R* ^*l* − *ω*+1^ with weight *W*_*c*_^*j*^ is constructed by the following formula:

(8) $$\begin{array}{c} c^{j}=\left[c_{1}^{j},c_{2}^{j},\ldots ,c_{i}^{j},\ldots ,c_{l-\omega +1}^{j}\right]. \end{array}$$

Information about platform users, subsystem connection configuration, XML data format, and teaching resource retrieval are the main components of the basic Japanese teaching resource database. Students' learning is centered on the knowledge points in instructional materials, which are also a key vehicle for reflecting the unique qualities of each student. The Arduino device identification program is used by students as they learn. It is based on CNN. Learners are informed of the names of the identified devices by the identification program, and learning materials, including text and video resources, are pushed to them that are pertinent to the devices. As instructional resources generally occupy more storage space, this paper adopts cloud storage mode. The main content stored in the resource table is the storage path of instructional resources uploaded by administrators and teachers. In addition to the storage path of the resource, the size of the resource, the query and comment permission of the resource are also saved in the table. The resource table is shown in Table 1.

RETRACTED

Because the level of students' cognitive ability is constantly improving and changing with the deepening of study, only real-time feedback and updating of students' cognitive ability can truly realize the recommendation of resources that are compatible with the real level. The content of this basic Japanese teaching resource database is constantly updated and improved, carefully selected by Japanese teachers, and can be directly linked with Japanese learning websites and Japanese exhibitions, further enriching students' autonomous learning resources.

## 4. Result Analysis and Discussion

The data in this study are randomly dispersed, with each data sample having the same likelihood of being either training data or testing data. The data are separated into training data sets and testing data sets in accordance with a specific proportion. The simulation experiment from this chapter is performed in MATLAB in this publication. The server side of this system's test environment consists of the following components: the Windows Server operating system, the SQL SERVER database management system, and the Net Framework. During the model's training phase, its parameters are iteratively adjusted and optimized. This process continues until either the output data value converges and tends to a stable state, the model training is complete, or the specified number of iterations has been reached. The classification of images can now be done by acquiring and using a classification model.  Figure 3 shows several trainings of this network.

In this study, the modeling impact of the model is tested using two widely used assessment criteria: the pattern accuracy rate and the RMSE (Root mean square error) index. Among these, the following formula illustrates the computation formula for the pattern accuracy index:

(9) $$\begin{array}{c} \text{PMR}=\frac{\sum_{t=1}^{T}\sum_{i=1}^{M}I^{\left(t\right)}\left({\overset{⟶}{\alpha }}_{i}={\hat{\overset{⟶}{\alpha }}}_{i}\right)}{T*M}. \end{array}$$

Among them, $I^{\left(t\right)}\left({\overset{⟶}{\alpha }}_{i}={\hat{\overset{⟶}{\alpha }}}_{i}\right)$ indicates whether the ${\hat{\overset{⟶}{\alpha }}}_{i}$ estimated in the *t* th experiment is the same as the real value ${\overset{⟶}{\alpha }}_{i}$. If the same, the value of $I^{\left(t\right)}\left({\overset{⟶}{\alpha }}_{i}={\hat{\overset{⟶}{\alpha }}}_{i}\right)$ is 1, otherwise it is 0. *M* and *T* represent the number of experiments and the number of experiments, respectively. The formula for calculating the RMSE indicator is shown in the following formula:

(10) $$\begin{array}{c} \text{RMSE}=\sqrt{\frac{\sum_{t=1}^{T}\sum_{l=1}^{2^{k}}\sum_{j=1}^{N}{\left[P^{\left(t\right)}\left({\overset{⟶}{r}}_{j}=r|{\overset{⟶}{\alpha }}_{i}\right)-{\hat{P}}^{\left(t\right)}\left({\overset{⟶}{r}}_{j}=r|{\overset{⟶}{\alpha }}_{i}\right)\right]}^{2}}{2^{k}*T*M}}. \end{array}$$

Among them, $P^{\left(t\right)}\left({\overset{⟶}{r}}_{j}=r|{\overset{⟶}{\alpha }}_{i}\right)$ and ${\hat{P}}^{\left(t\right)}\left({\overset{⟶}{r}}_{j}=r|{\overset{⟶}{\alpha }}_{i}\right)$ represent the probability that the *t* th experimental estimate and the real attribute mode ${\overset{⟶}{\alpha }}_{i}$ score *r* in the *j* th question, respectively. The estimated value is closer to the real value if the model accuracy value is greater and the RMSE value is smaller; in other words, the smaller the error, the more accurate the modeling algorithm.

RETRACTED

Every step of the network structure in this paper will reduce the size of input images by convolution or pooling. This reduces the amount of computation needed to train and test a network, and at the same time makes the output more general. In this chapter, 10%, 30%, 50%, 70%, and 90% of the data sets are selected as test data sets, and the results of the algorithms are compared when the data sparseness is different. The experimental results of pattern recognition rate values of different methods under various test data sets are shown in Figure 4. The experimental results of RMSE values of different algorithms are shown in Figure 5.

It can be seen that compared with other methods, the accuracy rate of this method is larger and the RMSE value is smaller.

Teachers' uploading resources is the embodiment of the data integration function provided by the platform. After logging in, teachers' users in the teachers' teaching management system can directly upload an instructional resource to the basic Japanese teaching resource management system. This function is the superior function embodiment of the data integration subsystem of the basic Japanese teaching resource pool sharing platform. The comparison results of the retrieval efficiency of different methods are shown in Figure 6.

The test environment is an intranet with a bandwidth of 100 M, and the query operation of a single resource is performed to ensure that the system performance is unaffected by the network speed. The experimental findings demonstrate the great retrieval efficiency of this technology. In this chapter, various approaches are contrasted in order to better test the impact of the model put forth in this study. The experimental results of precision and recall are shown in Table 2.

RETRACTED

In the adjusted network model of this paper, the image data is input from the bottom of the network, and after three convolution processing and corresponding pooling processing, the data is converted into a one-dimensional vector and input to the full connection layer, where finally, the test accuracy and error loss function values are output.  Figure 7 shows the accuracy of different network models.

It can be seen that the accuracy of this network model is high. This verifies the feasibility and effectiveness of the basic Japanese teaching resource database system based on DNN, thus achieving the expected effect of this paper. The experimental results of this chapter show that the precision rate and recall rate of the Japanese teaching resource database system constructed in this paper can reach about 93% and 94%, respectively. Its performance is superior to the traditional teaching resource system, and it can provide a high-quality instructional resource for basic Japanese teaching.

## 5. Conclusion

The social expectations for talent in Japanese education have not been met by traditional teaching methods. The use of network resources in contemporary Japanese instruction must be taken into consideration in order to broaden students' knowledge and raise their actual Japanese proficiency. The need, theoretical underpinnings, users, characteristics of the content, and issues that should be taken into consideration when building a basic Japanese teaching resource database are all covered in this essay. In light of the current, rapid development of information technology, this paper examines some issues with the creation of a database of Japanese teaching resources. Based on this, a fundamental DNN-based database of teaching resources for Japanese is built. The creation of a Japanese teaching resource database has made it possible to publish, search for, and maintain educational resources. The platform creates the operational form of seamless connection between various systems and executes the data integration function suggested in this paper. The experimental findings indicate that the precision rate and recall rate of the Japanese teaching resource database system developed in this paper can reach about 93 percent and 94 percent, respectively. Its performance is better than the conventional teaching resource system, and it can deliver high-quality teaching materials for the teaching of fundamental Japanese. We can further explore the new Japanese teaching mode, professional talent cultivation mode, and self-learning ability cultivation mode based on the professional teaching resource database mode by continuously developing and perfecting the professional teaching resource database. Contribute appropriately to developing highly qualified and creative higher-vocational talent that satisfies market demand.

RETRACTED

## Figures and Tables

**Figure 1:** DNN structure.

**Figure 2:** Arduino device identification and model training process.

**Figure 3:** Network training situation.

**Figure 4:** Comparison of pattern accuracy values of different methods under different test data set proportions.

**Figure 5:** Experimental results of RMSE values of different algorithms.

**Figure 6:** Comparison of the retrieval efficiency of different methods.

**Figure 7:** Comparison of the accuracy of different network models.

**Table 1:** Resource table settings.

Serial number	English name of the fields	Chinese name of the fields	Type and precision of fields	Data description
1	ZY_ID	Resource ID	Int	Not null
2	ZY_PATH	Resource path	Char (60)	Not null
3	ZY_SIZE	Resource size	Int	Not null
4	ZY_QUANXIAN	Resource authority	Char (10)	Null

**Table 2:** Experimental results of precision and recall of different algorithms.

Algorithm	Precision ratio (%)	Recall ratio (%)
Ant colony algorithm	84.21	85.34
K-Means algorithm	85.46	86.71
BP network algorithm	88.46	89.07
Algorithm in this paper	93.21	94.32

## Data Availability

The data used to support the findings of this study are available from the corresponding author upon request.
